The article "Clinical Impact of De-Regulated Notch-1 and Notch-3 in the Development and Progression of HPV-Associated Different Histological Subtypes of Precancerous and Cancerous Lesions of Human Uterine Cervix" was retracted in 2022. Reasons: errors in the images; duplicated images; unreliable results or conclusions.

# Clinical Impact of De-Regulated Notch-1 and Notch-3 in the Development and Progression of HPV-Associated Different Histological Subtypes of Precancerous and Cancerous Lesions of Human Uterine Cervix

**DOI:** 10.1371/journal.pone.0098642

**Published:** 2014-06-06

**Authors:** Richa Tripathi, Gayatri Rath, Poonam Jawanjal, Shweta Sharma, Pallavi Singhal, Suresh Bhambhani, Showket Hussain, Mausumi Bharadwaj

**Affiliations:** 1 Division of Molecular Genetics & Biochemistry, Institute of Cytology and Preventive Oncology (ICPO), ICMR, Noida, India; 2 Department of Anatomy, VMMC & Safdarjang Hospital, New Delhi, India; 3 Division of Pathology, Institute of Cytology and Preventive Oncology (ICPO), ICMR, Noida, India; Rajiv Gandhi Centre for Biotechnology, India

## Abstract

**Background:**

Cervical cancer is the leading cause of cancer related deaths among women in India. Limited reports are available for Notch-1 and Notch-3 protein in cervical carcinoma, which play crucial role in cell proliferation, differentiation, and apoptosis.

**Methods:**

This study was designed to evaluate the role of Notch-1 and Notch-3 with context to HPV infection in cervical carcinoma. A total of 168 tissue biopsy samples comprising of tumor specimens (n = 98), precancer (n = 30) and non-neoplastic cervical tissues (n = 40) were screened for HPV infection by PCR and expression of Notch-1 and Notch-3 protein by Immunohistochemistry and Immunoblotting.

**Results:**

80% (24/30) were found to be positive for HPV in precancer and 86.7% (85/98) in cancer patients. Notch-1 expression of precancer and cancer cases was found to be significantly down-regulated with severity of disease in nuclear (3.43±0.29; 2.04±0.19, p = 0.0001, p = 0.0001) and cytoplasm (3.07±0.29; 2.29±0.17, p = 0.0001, p = 0.0001) obtained from different stages as compared to normal cervix tissue (5.40±0.19, 4.97±0.15; p<0.001; p<0.001). However, Notch-3 expression of above cases was significantly up-regulated with severity of disease and showed intense nuclear (4.17±0.39; 4.74±0.18, p = 0.0001, p = 0.0001) and cytoplasm (3.67±0.36; 4.48±0.18, p = 0.0001, p = 0.0001) of different stages as compared to normal cervix tissue (0.95±0.20, 0.70±0.20; p<0.001; p<0.001) respectively.

**Conclusions:**

These findings suggest that Notch-1 and Notch-3 may play an important role with synergistic effect of HPV in regulating development and proliferation of cervical cancer through the deregulation of Notch signalling. This study also shows the clinical utility of both proteins which may be used as predictable biomarkers in diagnosing different histological sub-types of HPV associated cervical cancer. Nevertheless, abnormal activation of this pathway may provide legitimate targets for cervical cancer therapy.

The article "Clinical Impact of De-Regulated Notch-1 and Notch-3 in the Development and Progression of HPV-Associated Different Histological Subtypes of Precancerous and Cancerous Lesions of Human Uterine Cervix" was retracted in 2022. Reasons: errors in the images; duplicated images; unreliable results or conclusions.

## Introduction

Cervical cancer which was the second most common female cancer worldwide in 2008 [1] is now the fourth most common cancer affecting women worldwide, after breast, colorectal, and lung cancers with an incidence of about 528 000 new cases every year [2]. It is also the fourth most common cause of cancer death (266 000 deaths in 2012) in women worldwide [2]. This shows that the early cancer detection of cervical cancer worldwide using newer diagnostic modalities has improved the clinical outcome by detecting the disease at an early stage and thus minimizing the morbidity and improving survival rate. Over 80% of the cervical cancer present is at a fairly advanced stage. Almost 70% of the global burden falls in areas with lower levels of development and more than one fifth of all new cases are diagnosed in India [2] due to lack of screening that allows detection of pre-cancerous and early stage cervical cancer. Therefore, in India, this is still leading cancer among rural women.

Histologically, cervical cancer progresses from normal epithelium through a series of well defined precancer lesions referred to as cervical intraepithelial neoplasia (CIN) [1], [3]. It is suggested that HPV infection particularly HPV type 16 and 18 may be a causative factor, but infection alone is not sufficient to generate the full blown malignant phenotype. Also, the majority of HPV infections are subclinical; therefore, only a small number of carcinogenic HPV infections lead to cervical cancer development [4]. Thus, a major aspect of cervical cancer research is to identify other host factors, including alterations in signalling pathways that are involved in malignant transformation of cervical cells, which may predict the outcome of cervical cancer.

The Notch Signalling pathway is a complex transmembrane signalling pathway in higher eukaryotes that is involved in cell fate determination during development [5], [6]. The mammalian Notch genes (Notch-1, Notch-2, Notch-3, and Notch-4) encode 300 kDa single pass transmembrane receptors, which play important roles in a diverse group of developing tissues [6]. Binding of one of the Notch ligands, which include Delta1, Jagged-1, and Jagged-2, leads to a complex cleavage and activation of Notch proteins [6], [7]. The released and activated COOH-terminal fragment of Notch intracellular domain (NICD) translocates to the nucleus, in which it interacts with the transcription factor CBF1 (RBPjk) to transactivate target genes including HES-1[6]. The Notch gene is abnormally activated in tumorigenesis and can be either oncogenic or antiproliferative, and the function is context dependent [8].

The article "Clinical Impact of De-Regulated Notch-1 and Notch-3 in the Development and Progression of HPV-Associated Different Histological Subtypes of Precancerous and Cancerous Lesions of Human Uterine Cervix" was retracted in 2022. Reasons: errors in the images; duplicated images; unreliable results or conclusions.

Up-regulated expression of components of Notch is also related to many malignant tumors [9], [10]. Several studies showed that Notch-1 plays a significant role in acute T-cell lymphoblastic leukaemia, breast cancer, choriocarcinoma [11]–[13]. Transgenic mice that overexpress the NICD of Notch-3 in lung cancer and in mammary glands developing mammary tumors, suggesting the transforming potentials of Notch-3 in vivo [8], [14]. Notch-3 might also play important role for the proliferation and survival of ovarian and pancreatic cancer [15]–[16] but the exact mechanism is not clear. In addition, it is suggested that Notch signalling may be involved in neoplastic transformation in cervical carcinoma [17]. Oncogenic cooperation during Notch induced solid tumorigenesis has been reported. Cooperation between Notch and viral oncoproteins, such as simian virus 40 (SV40) largeT, adenovirus E1A and human papilloma virus (HPV) E6/E7 also contribute to tumorigenesis [13]. In the view of above, we measured both Notch-1 and Notch-3 expression levels in HPV associated various phases of tumor progression in the cervical epithelium, ranging from normal epithelium through low and high grades of squamous intraepithelial lesions (precancer) and invasive cervical cancer tissues to determine their role in this cancer.

## Material and Methods

### Ethics statement

All the patients included in our study had no family history of ISCC (Invasive squamous cell carcinoma) or any other disease and were not treated with chemotherapy prior to tumor removal. The study was approved by the research and ethics committee of Institute of Cytology and Preventive Oncology (ICPO)-ICMR, India. Written informed consent was obtained from all the subjects included in the study.

### Tissue specimens

A total of 168 biopsy tissue samples were obtained from the Department of Obstetrics and Gynecology at Safdarjang Hospital and Lok Nayak Jaiprakash hospital, New Delhi: 98 cervical squamous cell carcinomas, 30 precancer (19 CIN1, 03 CIN2 and 08 CIN3) and 40 from normal controls (UV-prolapse tissues, non-neoplastic). The clinico-pathological parameters of patients were collected as described by Bahnassy et al 2006 [18]. Tumor staging was performed according to the International Federation of Gynecology and Obstetrics (FIGO) classification [19]. Histo-pathological grades and clinical staging were evaluated according to standard criteria by two pathologists independently. Tissue samples were divided into two parts: one part was sent to histopathological diagnosis and other half was stored in −70°C for molecular investigations.

### Immunohistochemistry

Sections (5 µm) of formalin-fixed, paraffin-embedded ISCC specimens were mounted on poly-L-lysine (Sigma, St. Louis, MO, USA) coated slides and processed for conventional histological assessment by H&E staining and Immunohistochemistry (IHC) after de-waxing and then dehydrating. Antigen retrieval treatment was done in citrate buffer in microwave and then cooled for 20–30 min. After washing in 0.01M Tris-buffered saline (pH 7.4), sections were incubated with 1% BSA followed by overnight incubation at 4 C with primary polyclonal anti-human antibody of Notch-1 and Notch-3 (ab 8925, ab23426 Abcam) at a dilution of 1∶200 and 1∶500 respectively. An EnVision+System peroxidase kit (DAKO, Carpinteria, CA) was used for staining. Sections were then counterstained with Mayer's haematoxylin solution, dehydrated in ascending concentrations of ethanol (30% to 100%), cleared in xylene and mounted with DPX. For each target staining, all slides were processed at the same time. The stained tissue slides were examined under an Olympus microscope (model BX-51, Olympus America, Inc., Melville, NY) with ‘‘Olysia Bio-report’’ software linked with a personal computer. The primary antibody was replaced with isotype-specific IgG as a negative control.

The article "Clinical Impact of De-Regulated Notch-1 and Notch-3 in the Development and Progression of HPV-Associated Different Histological Subtypes of Precancerous and Cancerous Lesions of Human Uterine Cervix" was retracted in 2022. Reasons: errors in the images; duplicated images; unreliable results or conclusions.

### Scoring of Immunohistochemical staining

IHC results for Notch-1 and Notch-3 proteins have followed the scoring criterion indicated by Tripathi et al. 2010 [20]. Briefly, protein expression was semi quantified with regard to the intensity of cell staining graded as 0–3 ‘0’ for negative staining if there is total absence; score of ‘1’ for weak; ‘2’ for moderate and ‘3’ for intense positive staining), as well as to the percentage (ranging from 0 to 100%) of positive stain cells of any intensity ranging from 1 to 4+ as 0–10% = 0; 10–30% = 1; 30–50% = 2; 50–70% = 3 and 70–100% = 4. Finally, a total score was obtained by adding the score of percentage positivity and intensity.

### Immunoblotting

Protein extracts from all cervical tissues (precancer, cancer and normal control) were prepared and immunoblotting was done according to previos studies from our laboratory [21]–[23]. Polyclonal anti-human antibodies of Notch-1 and Notch-3, β-actin (rabbit monoclonal β-actin antibody (1∶2000, Abcam) and diluted (1∶4000 in BSA) secondary antibody HRP-conjugated rabbit anti-IgG (Abcam,) were used in this study. The bands were visualized using the Luminol based Enhanced chemiluminescence detection kit (Santa Cruz Biotech, USA). The expression levels of Notch-1 and Notch-3 were evaluated by densitometry using Alpha Digidoc version 4.1.0 (Alpha Innotech Corporation, IL) on a scale of 0–255 and the averaged pixel values were re-grouped for analysis on an arbitrary scale as strong = >50%; medium = 10–50%; weak = 1–10% and nil/not detectable as described previously [21]–[23]. The expression of Notch-1 and Notch-3 in tumor tissue was determined by quantitating and comparing it with their expression in normal tissues.

The article "Clinical Impact of De-Regulated Notch-1 and Notch-3 in the Development and Progression of HPV-Associated Different Histological Subtypes of Precancerous and Cancerous Lesions of Human Uterine Cervix" was retracted in 2022. Reasons: errors in the images; duplicated images; unreliable results or conclusions.

### Genomic DNA isolation

DNA was isolated from all the tissue biopsies by standard proteinase K digestion and phenol chloroform method routinely followed in our laboratory [22], [23]. Both the quality and integrity of genomic DNA were checked spectro-photometrically and on 1% agarose gel.

### HPV detection and HPV typing

All DNA samples were tested by duplex PCR assay using housekeeping human β-globin gene and consensus sequence primers, directed to a conserved L1 gene of HPV genome. This was done in the same PCR reaction in order to exclude false negative and false positive results according to the previous study from our laboratory [23] and hence able to detect all mucosal HPV types. For the distinction of HPV types, we used specific pair of primers for HPV-16 and HPV-18. The methodology for isolated DNA amplification by PCR along with the pair of primers used for β-globin, L1, HPV-16 and for HPV-18 was described by Singh et al., 2013. PCR product was further visualized on ethidium bromide stained 2% agarose gel. In order to avoid false positivity or false negative results, every PCR reaction included positive and negative controls. Furthermore, all HPV positive/negative samples were repeated in a separate PCR run in triplicate. DNA extraction, PCR reagent preparation, amplification, and amplicon analysis were performed in separate rooms. Disposable aeroguard pipette tips were used throughout the experiment. In addition, all positive samples were repeated in a separate PCR run and all were reproducible. Strict laboratory precautions and control measures were followed to avoid cross-contamination with amplicons and carry-over in the PCR assay [24].

### Statistical Analysis

Statistical analysis was carried out using statistical software SPSS 11.0. The analysis of expression of Notch-1 and Notch-3 proteins and correlation of their expression patterns in precancer and cancer cases with the clinico-pathological parameters of the patients was evaluated by Chi Square test. Interprotein correlation was done using Spearman correlation test. p≤0.05 was regarded as statistically significant.

## Results

### Expression profile of Notch-1 and Notch-3 protein in Precancerous and cancerous lesions of human cervix by Immunohistochemistry

We observed differential expression patterns of Notch-1 and Notch-3 protein in cervical precancer and cancer cases of different stages as compared to normal controls.

The article "Clinical Impact of De-Regulated Notch-1 and Notch-3 in the Development and Progression of HPV-Associated Different Histological Subtypes of Precancerous and Cancerous Lesions of Human Uterine Cervix" was retracted in 2022. Reasons: errors in the images; duplicated images; unreliable results or conclusions.

### Notch-1

A significant down-regulation of Notch-1 expression was observed in both nuclear (3.43±0.29; 2.04±0.19, p = 0.0001, p = 0.0001) and cytoplasm (3.07±0.29; 2.29±0.17, p = 0.0001, p = 0.0001) of precancer and cancer as compared to normal cervix tissue (5.40±0.19, 4.97±0.15; p<0.001; p<0.001) (Figure-1B-F). But, its localization on the cell membrane of epithelial cells was found to be increased (1.13±0.18; 1.46±0.14) in both as compared to normal cervix tissues (0.35 ±0.12; p = 0.010) (Table-1). Overall, 13.3% (4/30) of precancer tissues and 20.4% (20/98) of ISCC tissues expressed significant loss of cytoplasmic and nuclear Notch-1 protein expression (Table-2). Interestingly, the expression pattern of Notch-1 protein was lower than the basal level in LSIL (CIN1) which further significantly reduced in HSIL (CIN2/3, p = 0.0001, Table-1).

**Figure 1:** Immuno-histochemical analysis of Notch-1 and Notch-3 showing expression pattern of Notch-1 and Notch-3 in normal, precancerous and cancer tissues of uterine cervix. (**A**) Negative control of Notch-1 in normal tissue, 200X. (**B**) Intense nuclear, cytoplasmic expression and loss of membranous expression of Notch-1 in normal cervix, 200X. (**C**) Moderate nuclear expression of Notch-1 in precancrous tissue, 200X. (**D**) Negative control (ISCC, 200X). (**E**) Mild cytoplasmic localization and loss of nuclear Notch-1 in ISCC, 200X. (**F**) Membranous positive and loss of nuclear expression of Notch-1 in ISCC, 400X. (**G**) Negative control of Notch-3, 200X. (**H**) Cytoplasmic localization and loss of nuclear Notch-3 in normal cervix, 200X. (**I**) Cytoplasmic and nuclear localization of Notch-3 in precancer, 200X. (**J**) Negative control of Notch-3 (ISCC, 200X). (**K**) Cytoplasmic and Nuclear localization And loss of membranous Notch-3 in ISCC, 200X as indicated in Materials and Methods section. (**L**, **M**) Bar graph showing distribution of total scores of Notch-1 and Notch-3 protein in Normal cervix, Precancer and Invasive squamous cervical carcinoma (ISCC) tissues. The vertical axis shows the total Immunostaining score (cytoplasmic or nuclear respectively), obtained as described in the Methods section. (**N**) Western blots showing expression pattern of Notch-1 and Notch-3 protein during the progression of cervical cancer. Protein extracts from cervical tumor biopsies as well as normal tissues were separated in 10% SDS-PAGE and detected by specific antibodies of Notch-1 and Notch-3 protein. All the blots were stripped and reprobed for β-actin levels to confirm equal loading and the quantitation of bands was performed densitometrically as indicated in Materials and Methods section.

The article "Clinical Impact of De-Regulated Notch-1 and Notch-3 in the Development and Progression of HPV-Associated Different Histological Subtypes of Precancerous and Cancerous Lesions of Human Uterine Cervix" was retracted in 2022. Reasons: errors in the images; duplicated images; unreliable results or conclusions.

**Table 1:** Total score (Intensity score + Percentage positivity, Mean ± S.E) of Notch-1 and Notch-3 expression in normal, precancerous and cancer tissues.

Cases	Notch-1 (Total Score, Mean ± S.E)				Notch-3 (Total Score, Mean ± S.E)			
	Cyto (C)	Nuclear (N)	C+N	Membranous	Cyto (C)	Nuclear (N)	C+N	Membranous
Normal	4.97±0.15	5.40 ±0.19	5.19±0.16	0.35 ±0.12	0.95±0.20	0.70±0.20	0.82±0.19	2.28 ±0.24
LSIL	3.32±1.4	3.63±1.38	3.47±1.37	1.06±1.0	4.11±1.8	3.91±2.2	3.4±2.0	1.09±1.3
p-value	*0.0001	*0.0001	*0.0001	*0.002	*0.0001	*0.0001	*0.0001	*0.01
(LSIL Vs Normal)	(p<0.001)	(p<0.001)	(p<0.001)		(p<0.001)	(p<0.001)	(p<0.001)	
HSIL	2.64±1.96	3.09±1.9	2.86±1.9	1.09± 1.04	2.9±2.1	4.32±2.1	4.2±1.8	1.0±1.1
p-value	*0.0001	*0.0001	*0.0001	*0.010	*0.0001	*0.0001	*0.0001	*0.13
HSIL Vs Normal	(p<0.001)	(p<0.001)	(p<0.001)		(p<0.001)	(p<0.001)	(p<0.001)	
Total Pre-cancer (LSIL+ HSIL)	3.07±0.29	3.43±0.29 ▾	3.25±0.2 ▾	1.13±0.18▴	3.67±0.36	4.17 ±0.39 ▴	3.91±0.35 ▴	1.07±0.22 ▾
Cancer	2.29±0.17	2.04±0.19▾▾	2.14±0.18▾▾	1.46±0.14 ▴	4.48±0.18	4.74±0.18▴▴	4.61±0.16▴▴	0.92±0.12▾▾
p-value	*0.0001	*0.0001	*0.0001	*0.010	*0.0001	*0.0001	*0.0001	*0.01
(Total precancer Vs Normal)	(p<0.001)	(p<0.001)	(p<0.001)		(p<0.001)	(p<0.001)	(p<0.001)	
p-value	*0.0001	*0.0001	0.0001	0.0001	*0.0001	*0.0001	0.0001	*0.0001
(cancer Vs. normal)	(p<0.001)	(p<0.001)	(p<0.001)		(p<0.001)	(p<0.001)	(p<0.001)	

p-values are calculated using the chi-square test.

* p≤0.05 was considered significant.

▾ Downregulation;^▴^Upregulation.

**Table 2:** Positive percentage of Notch-1 and Notch-3 expression in normal, precancerous and cancer tissues.

Cases	Notch-1						Notch-3					
	Cyto		Nuclear		Cyto +Nuclear		Cyto		Nuclear		Cyto +Nuclear	
	(-)	(+)	(-)	(+)	(-)	(+)	(-)	(+)	(-)	(+)	(-)	(+)
	n(%)	n(%)	n(%)	n(%)	n(%)	n(%)	n(%)	n(%)	n(%)	n(%)	n(%)	n(%)
Normal (n = 40)	10(25)	30(75)	05(12.5)	35(87.5)	10(25)	30(75)	33(82.5)	07(17.5)	35(87.5)	5(12.5)	34(85)	06(15)
Precancer (n = 30)	25(83)	05(16.7)	25(83.3)	5(16.7)	26(86.7)	4(13.3)	07(23.3)	23(76.7)	05(16.7)	10(25)	04(13.3)	26(86.7)
ISCC (n = 98)	83(84.7)	15(15.3)	80(81.6)	18(18.4)	78(79.6)	20(20.4)	16(16.3)	82(83.7)	15(15.3)	83(84.7)	14(14.3)	84(85.7)
p-value	*0.0001		*0.0001		*0.0001		*0.0001		*0.0001		*0.0001	

p-values are calculated using the chi-square test. * p≤0.05 was considered significant.

### Notch-3

A significant up-regulation of Notch-3 expression was observed in nuclear (4.17±0.39; 4.74±0.18, p = 0.0001, p = 0.0001) and cytoplasm (3.67±0.36; 4.48±0.18, p = 0.0001, p = 0.0001) of precancer and cervical cancer of different stages as compared to normal cervix tissue (0.95±0.20, 0.70±0.20; p<0.001; p<0.001) respectively (Table-1, Figure-1H-K). But, its localization on the cell membrane of epithelial cells was found to be decreased (1.07±0.22; 0.92±0.12) in precancer and cancer as compared to normal cervix tissues (2.28±0.24; p = 0.001) (Table-1). Overall, 86.7% (26/30) of precancer and 85.7% (84/98) of ISCC tissues showed significant cytoplasmic and nuclear Notch-3 positivity (Table-2). The expression pattern of Notch-3 protein was significantly higher than the basal level in LSIL (CIN1, p = 0.0001) which further increased in HSIL (CIN2/3, p = 0.0001, Table-1). Although we could not observe any significant differences between LSIL and HSIL statistically (p = 0.55).

The article "Clinical Impact of De-Regulated Notch-1 and Notch-3 in the Development and Progression of HPV-Associated Different Histological Subtypes of Precancerous and Cancerous Lesions of Human Uterine Cervix" was retracted in 2022. Reasons: errors in the images; duplicated images; unreliable results or conclusions.

Figure-1L, M and Table-1 showed the total Immunostaining score distribution of nuclear and cytoplasmic Notch-1 and Notch-3 expression in cervix normal tissues, precancer and cervical carcinoma.

### Expression of Notch-1 and Notch-3 by Immunoblotting

We further validated our results by western blotting in all tissue biopsies comprising of precancer, cancer and normal controls using Notch-1 and Notch-3 antibody. We found the gradual decreased expression of Notch-1 (80kDa) and increased expression of Notch-3 (244 kDa) in precancer (P1, P2) and squamous cell cervical carcinoma (C1, C2) as compared to the normal tissues (N1, N2; Figure-1N). Hence, both Immunohistochemistry and Immunoblotting experiments corroborated well.

### Determination of potential of Notch-1 and Notch-3 expression to distinguish ISCC and Precancer from normal cervix tissue by Receiver Operating Characteristic (ROC) Curve analysis

#### Precancer

The values for area-under-the-curve (AUC) for cytoplasmic Notch-1 and Notch-3 were 0.82, 0.85 and for nuclear Notch-1 and Notch-3 were 0.82, 0.87 respectively. The sensitivity and specificity for cytoplasmic Notch-1 and Notch-3 were 99%, 95%; 76.7%, 82.5% respectively. Similarly, for nuclear Notch-1 and Notch-3 these were 99%, 95%; 83%, 75% respectively (Figure-2A, C; Table- S1, S2).

**Figure 2:** (A-D) Receiver operating characteristic curves of Notch-1(A, B) and Notch-3(C, D, nuclear and cytoplasmic) in normal vs. precancer (A, C) and ISCC (B, D). Blue line shows ROC analysis for cytoplasmic Notch-1/Notch-3. Green line shows ROC analysis for nuclear Notch-1/Notch-3 respectively. Y-axis of the plot shows true-positive fraction and X-axis shows false positive fraction.

#### Invasive Squamous Cell Carcinoma (ISCC)

The values for area-under-the-curve (AUC) for cytoplasmic Notch-1 and Notch-3 were 0.90, 0.91 and for nuclear Notch-1 and Notch-3 were 0.87, 0.93 respectively. The sensitivity and specificity for cytoplasmic Notch-1 and Notch-3 were 84.7%, 87.5%; 83.7%, 82.5% respectively. Similarly, for nuclear Notch-1 and Notch-3 these were 81.6%, 75%; 84.7%, 87.5% respectively (Figure-2B, D; Table- S1, S2).

The article "Clinical Impact of De-Regulated Notch-1 and Notch-3 in the Development and Progression of HPV-Associated Different Histological Subtypes of Precancerous and Cancerous Lesions of Human Uterine Cervix" was retracted in 2022. Reasons: errors in the images; duplicated images; unreliable results or conclusions.

### Correlation among Notch-1 and Notch-3 expression with clinico-pathological parameters of ISCC

We observed that 12.3% and 89.2% of Notch-1 and Notch-3 expression were found to be associated with tumor vaginal involvement respectively (p = 0.03; 0.03). Notch-1 also showed 12.2% of its expression with tumor size (p = 0.05) and 89.2% of Notch-3 showed its association with lymph node metastasis (p = 0.03).

Cytoplasmic, nuclear and total Notch-1 had lower and Notch-3 had higher percentage of (3.8%, 5.8%, 5.8%; 97%, 96.2%, 98.1%) moderately and poorly differentiated ISCC as compared to well differentiated ISCC (28.3%, 32.6%, 32.6%, p = 0.001; 67.4%, 71.7%, 71.7%, p = 0.001) respectively. Similarly, nuclear or total Notch-1 and Notch-3 showed 12.3% and 85.4% of progressed FIGO stage (III+IV) and 30.3% and 75% of FIGO stage-I+II (p = 0.03, p = 0.03; Table-3, 4).

**Table 3:** Analysis of Notch-1 protein expression in ISCC and its correlation with demographic and clinico-pathological parameters.

Parameters		Total No.	Notch-1 (Cyto)		p-value	Notch-1 (Nuclear)		p-value	Notch-1 (Cyto+ Nucl)		p-value
		N	- (%)	+(%)		- (%)	+(%)		- (%)	+(%)	
Age	<50	83	23(27.7)	60(72.3)	0.33	23(27.7)	60 (.5)	0.33	68(81.8)	15(18)	0.61
	≥ 50	15	06(40)	09(60)		05(33.3)	10(66.6))		12(80)	3(20)	
Gravidity	<3	16	14(87.5)	02(12.5)	0.73	14(87.5)	02(80.5)	0.50	13(81.3)	3(18.8)	0.85
	≥3	82	69(84.1)	13(15.9)		66(80.5)	16(19.5)		65(79.3)	17(20.7)	
Parity	<3	18	14(77.8)	04(86.3)	0.36	14(77.8)	04(22.2)	0.64	15(83.3)	3(16.7)	0.66
	≥3	80	69(22.2)	11(13.8)		66(82.5)	14(17.5)		63(78.8)	17(21.3)	
Smoking	No	63	51(81)	12(91.4)	0.16	50(79.4)	13(20.6)	0.43	50(79.4)	13(20.6)	0.49
	Yes	35	32(19)	03(8.6)		30(85.7)	05(14.3)		30(85.7)	5(14.3)	
Tobacco	No	62	51(82.2)	11(17.7)	0.37	49(79)	13(21)	0.38	49(79)	13(21)	0.38
	Yes	36	32(88.9)	04(11.1)		31(26.1)	05(13.9)		31(86.1)	5(13.9)	
Tumor size	<4	16	11(68.8)	05(31.3)	*0.05	11(16.8)	05(31.3)	0.14	11(68.8)	5(31.3)	0.14
	≥4	82	72(87.8)	10(12.2)		69(84.1)	13(15.9)		69(84.1)	13(72.2)	
Vaginal Invo	No	33	26(78.8)	07(21.2)	0.24	23(69.7)	10(30.3)	*0.03	23(69.7)	10(30.3)	*0.03
	Yes	65	57(87.7)	08(12.3)		57(87.7)	08(12.3)		57(87.7)	8(12.3)	
Grades	G1	46	33(71.7)	13(28.3)	*0.001	31(67.4)	15(32.6)	*0.001	31(67.4)	15(32.6)	*0.001
	G1+G2	52	50(96.2)	02(3.8)		49(94.2)	03(5.8)		49(94.2)	3(5.8)	
Lymph Nodes	No	33	28(84.8)	05(15.2)	0.97	27(81.8)	06(18.2)	0.97	27(81.8)	6(18.2)	0.97
	Yes	65	55(84.6)	10(15.4)		53(81.5)	12(18.5)		53(81.5)	12(18.5)	
FIGO Stage	I + II	33	26(78.8)	07(87.7)	0.24	23(69.7)	10(30.3)	*0.03	23(69.7)	10(30.3)	*0.03
	III+IV	65	57(21.2)	08(12.3)		57(87.7)	08(12.3)		57(87.7)	8(12.3)	

*p≤0.05 is considered as significant.

The article "Clinical Impact of De-Regulated Notch-1 and Notch-3 in the Development and Progression of HPV-Associated Different Histological Subtypes of Precancerous and Cancerous Lesions of Human Uterine Cervix" was retracted in 2022. Reasons: errors in the images; duplicated images; unreliable results or conclusions.

**Table 4:** Analysis of Notch-3 protein expression in ISCC and its correlation with demographic and clinico-pathological parameters.

Parameters		Total No.	Notch-3 (Cyto)		p-value	Notch-3 (Nuclear)		p-value	Notch-3(Cyto+ Nuc)		p-value
		N	- (%)	+(%)		- (%)	+(%)		- (%)	+(%)	
Age	<50	16	04(25)	12(75)	0.660	4(25)	12(75)	0.66	4(25)	12(75)	0.66
	≥ 50	82	25(30.5)	57(69.5)		25(30.5)	57(69.5)		25(30.5)	57(69.5)	
Gravidity	<3	16	2(12.5)	14(17.1)	0.65	2(12.5)	14(87.5)	0.73	2(12.5)	14(16.7)	0.82
	≥3	82	14(87.5)	68(82.9)		13(15.9)	69(84.1)		2(14.6)	70(85.4)	
Parity	<3	18	5(27.8)	13(72.2)	0.14	05(27.8)	13(72.2)	0.10	5(27.8)	13(72.2)	0.10
	≥3	80	11(13.8)	69(86.3)		10(12.5)	70(87.5)		9(11.3)	70(87.5)	
Smoking	No	63	12(19)	51(81)	0.16	14(22.2)	49(77.8)	*0.03	13(20.6)	50(79.4)	*0.01
	Yes	35	03(8.6)	32(91.4)		02(5.7)	33(94.3)		01(2.9)	34(97.1	
Tobacco	No	62	10(16.1)	52(83.9)	0.76	14(22.6)	48(77.4)	*0.02	12(19.4)	50(80.6)	0.06
	Yes	36	5(13.9)	31(86.1)		2(5.6)	34(94.4)		2(5.6)	34(94.4)	
Tumor size	<4	16	4(25)	12(75)	0.30	3(18.8)	13(81.3)	0.67	3(18.8)	13(81.3)	0.57
	≥4	82	12(14.6)	70(85.4)		12(14.6)	70(85.4)		11(13.3)	71(86.6)	
Vaginal Invo	No	33	7(21.2)	26(78.8)	0.24	09(27.3)	24(72.7)	*0.03	6(18.2)	27(81.8)	0.43
	Yes	65	8(12.3)	57(87.7)		7(10.8)	58(89.2)		8(12.3)	57(87.7)	
	G1	46	15(32.6)	31(67.4)	*0.001	13(28.3)	33(71.7)	*0.001	13(28.3)	33(71.7)	
	G1+G2	52	1(1.9)	51(97)		2(3.8)	50(96.2)		1(1.9)	51(98.1)	
Lymph Nodes	No	33	5(15.2)	28(84.8)	0.97	9(27.3)	24(72.7)	*0.03	7(21.2)	26(78.8)	0.16
	Yes	65	10(15.4)	55(84.6)		7(10.8)	58(89.2)		7(10.8)	58(89.2)	
FIGO Stage	I + II	16	7(21.2)	26(78.8)	0.24	4(25)	12(75)	*0.03	6(18.2)	27(81.8)	0.43
	III+IV	82	8(12.3)	57(87.7)		12(14.6)	70(85.4)		08(12.3)	57(87.7)	

*p≤0.05 is considered as significant.

### Prevalence of Human Papilloma Virus Infection in Precancer and Cervical Cancer

This study revealed 85% (109/128) of total (precancer and cancer) HPV-L1 positivity and 14.8% (19/128) of HPV-L1 negativity. Among them, 80% (24/30) of precancerous lesions and 86.7% (85/98) of tumor biopsies were infected with HPV. However, among HPV negative cases, majority of them were from precancerous lesions (20%) and 13.3% were from tumor biopsies which include 11% from Grade-I tumors and 2% from Grade-II+ Grade-III tumors.

Subsequent PCR based HPV typing using type specific primers revealed that a 96%(82/85) of HPV-L1 positive cervical tumors harbored high risk Human Papilloma virus (HR-HPV) type 16 however, 7.0%(6/85) of cancer ones were found to be infected with HPV-18 and 3.5% (03/85) of L1 positive cervical tumor cases showed co-infection with HPV type 16 and HPV type 18 (Figure-3B, C, D). Also, 5% (2/40) healthy controls were found to be HPV positive and all of them were infected with HPV type 16. Also, all precancerous HPV-L1 positive lesions were infected with HPV type 16 (Table-S3).

The article "Clinical Impact of De-Regulated Notch-1 and Notch-3 in the Development and Progression of HPV-Associated Different Histological Subtypes of Precancerous and Cancerous Lesions of Human Uterine Cervix" was retracted in 2022. Reasons: errors in the images; duplicated images; unreliable results or conclusions.

**Figure 3:** Detection of Human Papilloma virus genotypes 16 and 18 in precancer & cervical cancer patients by In vitro nucleic acid amplification test. (**A**) β-globin, 288bp (**B**) HPV-L1, 450bp (**C**) HPV-16, 217bp (**D**) HPV-18, 100bp as indicated in Materials and Methods section.

### Correlation among HPV and clinico-pathological parameters of ISCC

Analysis of HPV infection was correlated with clinico-pathological parameters (Table-5). Tumor vaginal involvement was found to be associated with 89.2% of HPV-16 (p = 0.03), tumor histopathological degree - moderately and poorly differentiated ISCC had higher percentage (94.2%) of HPV-16 positivity as compared to well differentiated ISCC (71.7%, p = 0.003) and 89.2% of HPV-16 with progressed FIGO stage (III+IV) and 79.2% in FIGO stage-I+II (p = 0.03). In the view of above, HPV-16 confirms its significant involvement with progression of cervical cancer.

**Table 5:** Analysis of HPV in ISCC and its correlation with clinico-athological parameters.

Clinico-pathological Parameters	Total No (N)	HPV-16			HPV-18			HPV overall positive		
		- (%)	+(%)	p-value	- (%)	+(%)	p-value	- (%)	+(%)	p-value
Tumor size										
<4	16	4(25)	12(75)	0.30	15(93.8)	1(6.3)	0.981	04(25)	12(75)	0.130
≥4	82	12(14.6)	70(85.4)		77(93.9)	5(6.1)		09(11)	73(89)	
Vaginal Involvement										
No	33	09(27.3)	24(72.7)	*0.03	31(93.9)	2(6.1)	0.98	08(24.2)	25(75.8)	*0.02
Yes	65	7(10.8)	58(89.2)		61(93.8)	4(6.2)		05(7.7)	60(92.3)	
Grade										
G1	46	13(28.3)	33(71.7)	*0.003	41(89.1)	5(10.9)	0.06	11(23.9)	35(76.1)	*0.003
G2+G3	52	3(5.8)	49(94.2)		51(98.1)	11(1.9)		2(3.8)	50(96.2)	
Lymph nodes										
No	33	06(18.2)	27(87.8)	0.72	33(100)	0(0)	0.07	06(18.2)	27(81.8)	0.30
Yes	65	10(15.4)	55(84.6)		59(90.8)	6(9.2)		07(10.8)	58(89.2)	
FIGO stage										
I+II	33	9(27.3)	24(72.7)	*0.03	31(93.9)	2(6.1)	0.98	8(24.2)	25(75.8)	*0.02
III+IV	65	7(10.8)	58(89.2)		61(93.8)	4(6.2)		5(7.7)	60(92.3)	

p-values are calculated using the chi-square test.

*p≤0.05 was considered significant.

### Impact of HPV infection on Notch-1 and Notch-3 protein in Precancerous and ISCC lesions

Correlation of HPV infection with Notch-1 and Notch-3 proteins in precancer and ISCC was done and shown in Table-6, 7, 8, 9, S4, S5. Our results showed that precancer patients which were HPV-16 negative showed 83.3% nuclear and cytoplsmic Notch-1 positivity (5 out of 6) and 50% nuclear and 33.3% cytoplasmic Notch-3 positivity. However, HPV-16 positive precancer cases does not show Notch-1 expression, however, these cases were significantly associated with 87.5% cytoplasmic Notch-3 (p = 0.005) and 91.7% nuclear Notch-3 (p = 0.01). In ISCC, total patients who were HPV negative showed 92.3% nuclear and 77% cytoplasmic Notch-1 positivity, however, these patients showed only 15.4% nuclear and cytoplasmic Notch-3 positivity. Among them, HPV-16 negative tumors showed 93.8% nuclear and 75% cytoplasmic Notch-1 positivity and 31.3% of nuclear and cytoplasmic Notch-3 positivity. Also, HPV-16 positive cervical carcinomas patients were observed to be associated with decreased cytoplasmic and nuclear Notch-1(3.7%, 3.7%, p = 0.0001, p = 0.0001) and with increased 93.9% of cytoplasmic Notch-3 and 95.1% of nuclear Notch-3. ISCC patients who were HPV-18 negative showed only 10.9% cytoplasmic Notch-1 positivity and 84.8% of nuclear and 82.6% of cytoplasmic Notch-3 positivity. HPV-18 positive patients was found to be significantly associated with increased Notch-1 expression levels (83.3%, 100%, p = 0.0001, p = 0.0001) respectively in precancer and cancerous lesions, however, HPV-18 was not found to be associated with Notch-3 expression levels in precancerous lesions and cancerous lesions. This supports the hypothesis that de-regulated Notch signalling may play a permissive or tumor promoting role in precancer and cervical carcinogenesis by synergizing with HPV-16 and HPV-18.

The article "Clinical Impact of De-Regulated Notch-1 and Notch-3 in the Development and Progression of HPV-Associated Different Histological Subtypes of Precancerous and Cancerous Lesions of Human Uterine Cervix" was retracted in 2022. Reasons: errors in the images; duplicated images; unreliable results or conclusions.

**Table 6:** Correlation of HPV infection with Notch-1 protein expression in precancer.

HPV		Cases	Notch-1 cyto (C)		p-value	Notch-1 nuc (N)		p-value	Notch-1 (C+N)		p-value
			-n(%)	+n(%)		-n(%)	+n(%)		-n(%)	+ n(%)	
HPV-16	No	06	1(16.7)	5(83.3)	*0.0001	1(16.7)	5(83.3)	*0.0001	1(16.7)	5(83.3)	*0.0001
	Yes	24	24(100)	0(0)		24(100)	0(0)		24(100)	0(0)	
HPV-18	No	30	25(83.3)	5(16.7)	-	25(83.3)	5(16.7)	-	25(83.3)	5(16.7)	-
	Yes	0	-	-		-	-		-	-	
HPV Overall positive	No	06	1(16.7)	5(83.3)	*0.0001	1(16.7)	5(83.3)	*0.0001	1(16.7)	5(83.3)	*0.0001
	Yes	24	24(100)	0(0)		24(100)	0(0)		24(100)	0(0)	

*p≤0.05 is considered as significant.

**Table 7:** Correlation of HPV infection with Notch-1 protein expression in ISCC.

HPV		Cases	Notch-1 cyto (C)		p-value	Notch-1 nucl (N)		p-value	Notch-1(C+N)		p-value
			-n(%)	+n(%)		-n(%)	+ n(%)		- n(%)	+n(%)	
HPV-16	No	16	04(25)	12(75)	*0.0001	01(6.3)	15(93.8)	*0.0001	2(11.8)	14(85)	*0.0001
	Yes	82	79(96.3)	03(3.7)		79(96.3)	03(3.7)		79(98)	03(3.7)	
HPV-18	No	92	82(89.1)	10(10.9)	*0.0001	80(87)	0(0)	*0.0001	80(87)	12(13)	*0.0001
	Yes	06	01(6.7)	05(83.3)		12(13.0)	06(100)		0(0)	6(100)	
HPV overall positive	No	13	03(23.1)	10(77)	*0.0001	1(7.7)	12(92.3)	*0.0001	01(7.7)	12(92.9)	*0.0001
	Yes	85	80(94.1)	05(5.9)		79(92.9)	06(7.1)		79(92.9)	06(7.1)	

*p≤0.05 is considered as significant.

The article "Clinical Impact of De-Regulated Notch-1 and Notch-3 in the Development and Progression of HPV-Associated Different Histological Subtypes of Precancerous and Cancerous Lesions of Human Uterine Cervix" was retracted in 2022. Reasons: errors in the images; duplicated images; unreliable results or conclusions.

**Table 8:** Correlation of HPV infection with Notch-3 protein expression in precancer.

HPV		Cases	Notch-3 cyto (C)		p-value	Notch-3 nucl (N)		p-value	Notch-3 (C+N)		p-value
			-n(%)	+ n(%)		- n(%)	+ n(%)		- n(%)	+n(%)	
HPV-16	No	06	4(66.7)	2(33.3)	*0.005	3(50)	3(50)	*0.01	2(33.3)	4(66.7)	*0.10
	Yes	24	3(12.5)	21(87.5)		2(8.3)	22(91.7)		2(8.3)	22(91.7)	
HPV-18	No	30	7(23.3)	23(76.7)	-	5(16.7)	25(83.3)	-	4(13.3)	26(86.7)	-
	Yes	0	-	-	-	-	-	-	-	-	
HPV Overall positive	No	6	4(66.7)	2(33.3)	*0.005	3(50)	3(50)	*0.01	2(33.3)	4(66.7)	*0.10
	Yes	24	3(12.5)	21(87.5)		2(8.3)	22(91.7)		2(8.3)	22(91.7)	

*p≤0.05 is considered as significant.

**Table 9:** Correlation of HPV infection with Notch-3 protein expression in ISCC.

HPV		Cases	Notch-3 cyto (C)		p-value	Notch-3 nuc (N)		p-value	Notch-3(C+N)		p-value
			- n(%)	+ n(%)		- n(%)	+ n(%)		- n(%)	+n(%)	
HPV-16	No	16	11(68.3)	5(31.3)	*0.0001	11(68.8)	5(31.3)	*0.0001	10(62.5)	6(37.5)	*0.0001
	Yes	82	5(6.1)	77(93.9)		4(4.9)	78(95.1)		4(4.9)	78(95.1)	
HPV-18	No	92	16(74)	76(82.6)	0.264	14(15.2)	78(84.8)	0.924	14(100)	8(84.8)	0.302
	Yes	06	0(0)	6(100)		1(16.7)	5(83.3)		0(0)	6(100)	
HPV overall positive	No	13	11(84.6)	2(15.4)	*0.0001	11(84.6)	2(15.4)	*0.0001	10(76.9)	3(23.1)	*0.0001
	Yes	85	5(5.9)	80(94.1)		4(26.7)	81(95.3)		4(4.7)	81(95.3)	

*p≤0.05 is considered as significant.

### Relationships between Notch-1 and Notch-3 expression in precancer and ISCC

The Spearman correlation test was carried out to identify the protein-protein inter-correlations in precancer and ISCC (Figure-S1). No association was observed in above two proteins in precancer patients. In ISCC patients, the significant negative associations were observed among cytoplasmic, nuclear and cyto+nuc Notch-1 and Notch-3 (r = −0.30, p  = 0.003; r = −0.28, p = 0.0004; r = −0.27, p  = 0.007) respectively (Figure-S1).

## Discussion

In India, cervical cancer is a leading cause of cancer related deaths in women, contributing approximately one fifth of the total cancer burden worldwide [2]. The progression of precancer of the uterine cervix to invasive cancer continues to remain an intensely studied problem in gynaecological pathology. Substantial decline in incidence and mortality of cervical cancer (2008–2012) in high-income countries such as the United States [25] have been attributed to its diagnosis at early stages and treatment of pre-invasive lesions. Conventionally, early detection of cervical cancer lesions is achieved by colposcopy and Papanicolaou smear test (or Pap test) which involves Liquid-based cervical specimen (LBC) in more than 90% of Pap tests [26]. In developed countries, proportion of women screened by Pap test is reported to vary from 68% to 84% [27]–[28] as compared to an appalling 2.6% to 5% in India [29].

The article "Clinical Impact of De-Regulated Notch-1 and Notch-3 in the Development and Progression of HPV-Associated Different Histological Subtypes of Precancerous and Cancerous Lesions of Human Uterine Cervix" was retracted in 2022. Reasons: errors in the images; duplicated images; unreliable results or conclusions.

Hence, these screening approaches may not be appropriate in middle and low-income countries like India as they are more expensive and not cost effective for mass screening where women living in low resource, medically underserved regions, training personnel such as cytotechnicians and pathologists and implementing continuous quality assurance procedures have proven difficulties. Also, socioeconomic status, access to care, and lack of health insurance coverage correlates with delay in diagnosis, advanced stage, and impaired survival. Almost 80% of the cervical cancer in India present to a tertiary care hospital at a fairly advanced stage, thereby, reducing the treatment options and survival rate [30], [31], [32]. Hence, research is needed to identify the optimal way of implementation of cervical cancer diagnosis and prevention in India, taking into account the cost and the human resources [33].

In addition to visual inspection methods (VIA) that are suitable for low resource settings, molecular-based HPV DNA testing have revolutionized in identifying women who are at risk for developing pre-invasive cervical lesions to invasive cancer with greater sensitivity as compared with Pap testing. It is important since majority of HPV infections are transient and asymptomatic and are undetectable by cytology or Visual inspection methods (VIA). HPV DNA testing not only identifies women with cervical disease but also those who are at risk for developing CIN within the next 3 to 10 years [34]. This is particularly important for developing countries that might not have sufficient resources to screen all women at 5 to 10 year intervals. Therefore, HPV molecular-based detection and genotyping technologies may offer an additional clinical advantage when screening for cervical cancer. Persistence infection with high-risk human papillomavirus (HR-HPVs) with constitutive expression of E6 and E7 viral oncogenes contributes to the development of cervical intraepithelial neoplasia (CIN), progression from CIN to cervical cancer and hence, is a necessary step for malignant transformation of cervical tissue [35]. Various reports have shown that in India, over 70% of cervical cancer cases harbor HPV infection and HPV-16 is the type exclusively prevalent in Indian women followed by HPV-18 [36]. India not only contains large geographical diversity but also has contrasting cultural variations and different religions that have been shown to influence the sexual behavior of women and their male partners, leading to differential acquisition of new HPVs [37]. In a National HPV mapping study in India using Southern blotting, the prevalence of HPV-16 was found to be highest in Chennai (88%) and lowest in Jammu and Kashmir (14.2%) [1], [38]. In the current report, all the cervical biopsies were screened for HPV infection by L1 consensus PCR and further sub-typing was done by using type specific primers for high risk HPV types 16 and 18. This study showed 85% (109/128) of total (precancer and cancer) HPV-L1 positivity. Among them, 80% (24/30) of precancerous lesions and 86.7% (85/98) of tumor biopsies were infected with HPV. Also, all of precancer and 96% (82/85) of HPV-L1 positive ISCC cases harbored high risk Human Papilloma virus (HR-HPV) type 16. None of precancer patient was found to be infected with HPV-18 however, 7.0% (06/85) of cancer ones were found to be infected with HPV-18. This is in agreement with the studies that showed that the prevalence of HPV type-16 in India is found to be exclusively very high [1], [39]. Epidemiological data have suggested approximately 10% of the healthy women have been found to harbor HPV infection [40] but in the present study we detect 5% of HPV infection in normal controls. This could be to the controls we collected may already cleared HPV infection. We also observed a significant association of HPV infection with vaginal involvement of tumor (p = 0.02), different pathological grades (p = 0.003) and FIGO stage (p = 0.02) of ISCC. This shows progressive involvement of HPV in the development of cervical cancer (from precancer to invasive cancer).

The article "Clinical Impact of De-Regulated Notch-1 and Notch-3 in the Development and Progression of HPV-Associated Different Histological Subtypes of Precancerous and Cancerous Lesions of Human Uterine Cervix" was retracted in 2022. Reasons: errors in the images; duplicated images; unreliable results or conclusions.

In this study, 14.8% (19/128) of HPV-L1 negativity was observed. However, majority (20%) of HPV negative cases were from precancerous lesions and 13.3% were from tumor biopsies which include 11% from Grade-I tumors and 2% from Grade-II+ Grade-III tumors. The reason behind the presence of HPV negative tumors could be explained on the basis of several lines reports world over who have demonstrated that the frequency of HPV infection in cervical cancer cases lies between 80–99% [36]. This clearly indicates the possible role of other independent risk factors including high parity, low socio-economic status, smoking, use of contraceptives, previous exposure to sexually transmitted diseases other than HPV and sexual behaviour of a woman's husband may be associated with cervical carcinoma. The hypothesis can be further strengthened by the fact that both experimental and epidemiological evidence has established high-risk human papillomavirus (HR-HPV) as the major etiological agent for the development of cervical cancer [1], [41]. However, cervical infection with HPV usually results in transient infection, with 70–90% of individuals demonstrating virus clearance within 12–24 months of detection. Persistent HPV infection in the remaining 10–30%, especially those with HR-HPV, may lead to the development of cervical intraepithelial neoplasia (CIN), a precursor of invasive carcinoma. Thus, HPV infection alone is not sufficient, but together with alterations in signalling pathways, environmental, host genetic and epigenetic factors may transform normal cervical cells into malignant cancer cells of uterine cervix [1], [42], [43]. Therefore, the activation of molecular pathways like Notch signalling may play central role in cervical cancer progression and biomarkers of such signalling pathway that could detect the disease early, predict aggressive behavior, and/or define molecular markers for more effective targeted therapy could offer newer insights to improve the existing therapeutic window [44].

The article "Clinical Impact of De-Regulated Notch-1 and Notch-3 in the Development and Progression of HPV-Associated Different Histological Subtypes of Precancerous and Cancerous Lesions of Human Uterine Cervix" was retracted in 2022. Reasons: errors in the images; duplicated images; unreliable results or conclusions.

The Notch signalling pathway is an evolutionarily conserved cell signalling pathway which plays a pivotal role in cell fate determination. De-regulated Notch signalling is oncogenic, inhibits apoptosis and promotes cell survival [45]. Aberrant Notch signalling is associated with several human diseases including cancers by altering the developmental state of a cell and consequently maintaining the cells in a proliferative or undifferentiated fate. Thus, Notch signalling plays a crucial role in tumor development by causing cells to adopt a proliferative cell fate [45].

Currently, Immunohistochemisrty (IHC) represents the most powerful tool for cervical cancer management which is also widely used in basic research to understand the distribution and localization of biomarkers that are differentially expressed proteins in cancer lesions. This, in turn, can provide information on the biological behaviour and prognosis of a tumor [46]. The combination of such diagnostic approaches along with combination of HPV DNA testing may represent the potential to further improve the detection of pre-invasive disease and thereby reduce the incidence of high-grade lesions compared with cytology testing alone.

In an attempt to elucidate the crucial role of Notch signalling in HPV mediated cervical cancer, the current study was designed to evaluate the expression of Notch-1 and Notch-3 proteins in precancer and ISCC specimens, and further to determine their involvement in the activation of the Notch signalling pathway. We observed down-regulation of Notch-1 in nuclear and cytoplasm of precancer and cervical cancer as compared to normal cervix tissue (<0.001; p<0.001) respectively. However, its expression decreases in ISCC (2.14±0.18) as compared to precancerous lesions (3.25±0.2). In precancerous lesions, the total positivity percentage of nuclear Notch-1 is found to be 16.7% (05/30) and in ISCC 18.4% (18/98), respectively. It appears that although there is little difference in the positivity percentage of Notch-1 in precancer and ISCC, its expression level was higher in precancerous lesions as compared to ISCC. Above results corroborates with Talora et al., 2002 [47] showing that precancer patients showed enhanced Notch-1 protein expression as compared to ISCC which showed its reduced levels.

The article "Clinical Impact of De-Regulated Notch-1 and Notch-3 in the Development and Progression of HPV-Associated Different Histological Subtypes of Precancerous and Cancerous Lesions of Human Uterine Cervix" was retracted in 2022. Reasons: errors in the images; duplicated images; unreliable results or conclusions.

We also analyzed the impact of HPV infection on loss of Notch-1 and observed that in precancerous lesions, nuclear Notch-1 expression was absent in HPV-16 positive cases and present (83.3%) only in HPV-16 negative ones. Similar results in ISCC patients were observed, that is, its expression was present in 93.8% of HPV-16 negatives and only 3.7% in HPV-16 positives. This supports the hypothesis that expression of Notch-1 in precancerous lesions, exerts specific protective effects against HPV-induced transformation through suppression of E6/E7 expression, and down-modulation of Notch-1 expression is likely to play an important role in late stages of HPV-induced carcinogenesis, suggesting a negative feedback between these viral oncogenes and Notch-1. Also, down-modulation of Notch-1 in ISCC is required for sustained HPV E6/E7 expression and HPV-16 induced transformation of malignant cells.

Notch-3 receptor is one of the mammalian Notch family receptors (Notch-1–4) which plays an important role in the regulation of cellular proliferation, differentiation, and apoptosis. In this study, the total positivity percentage of nuclear Notch-3 in precancerous lesions and in ISCC, was found to be 25% (10/30) and 84.7% (83/98) respectively. Also, over-expression of Notch-3 was observed in nuclear and cytoplasm of precancer and cervical cancer as compared to normal cervix tissue (p<0.0001, p<0.0001) respectively. Therefore, in cervical cancer cells that express Notch-3 may play two functional roles. First, Notch-3 serves as a receptor and after binding with its ligand stimulates adjacent tumor cells in a juxtacrine manner. Second, the intracellular domain of Notch-3 may trigger signalling pathway and promote tumor cell growth. This supports the hypothesis of an activation and deregulation of Notch signalling and shows that Notch signalling may provide a permissive environment for development of early pre-cancerous lesions which may lead to development and proliferation of cervical tumors and hence, it is one of the possible transducer of cervical carcinogenesis. Here, our results are in accordance with Yeasmin et al 2010 [17] partially who also showed an over-expression of Notch-3 in ISCC. However, we have extended our work with respect to HPV status. By analyzing the impact of HPV infection on this increase of Notch-3 expression, we found that in HPV-16 negative precancerous lesions and in ISCC, nuclear Notch-3 expression was decreased (33.3%, 31.3%) and in HPV-16 positive ones it was found to be increased (91.7%, 95.1%) respectively. It was observed that only Notch-3 was found to be significantly associated with HPV-16 in precancer (p = 0.0001) and both Notch-1 and Notch-3 with HPV infected ISCC (p = 0.0001, p = 0.0001). This up-regulated expression of Notch-3 in precancer and ISCC may trigger E6 and E7 oncoproteins of HPV which may promote tumor formation in precancer and late stages of cervical cancer. This shows that de-regulated signalling of above proteins indicates their possible involvement in establishment of HPV infection and persistence, suggesting that there may a complex interplay between Notch signalling and papillomaviruses in the context of development of cervical carcinogenesis. This study is also supported by Leong and Karson, 2006 [13] who discussed two mechanisms involved in Notch-induced oncogenesis in hematologic malignancies which include inhibition of apoptosis and induction of proliferation. These Notch proteins do not physically interact with each other, but may activate various signalling pathways to inhibit apoptosis and promote cell proliferation. Notch-3 can activate the PI3kinase-PKB/Akt pathway, a signalling cascade that is active in diverse cancers–and this along with the multifunctional HPV oncoproteins (E6 and E7) synergise with each other in tumorigenesis [48]. Above results showed that Notch receptors participate in the early and late stages of tumor progression and the expression of oncoproteins E6 and E7 is hypothesized to antagonize late stages of tumor progression.

The article "Clinical Impact of De-Regulated Notch-1 and Notch-3 in the Development and Progression of HPV-Associated Different Histological Subtypes of Precancerous and Cancerous Lesions of Human Uterine Cervix" was retracted in 2022. Reasons: errors in the images; duplicated images; unreliable results or conclusions.

In ISCC, significant negative associations were observed between nuclear and cytoplasmic expression of Notch-3 and nuclear, cytoplasmic localization of Notch-1 (r = −0.318, p = 0.001; r = −0.301, p = 0.003) respectively. Hence, Notch-3 and Notch-1 are inversely related to each other.

With respect to clinico-pathological parameters, nuclear Notch-1 was found to be significantly inversely associated with progressed tumor grade (p = 0.001), vaginal involvement of tumor (p = 0.03), progressed FIGO stage (p = 0.03) and with progressed tumor size (p = 0.05). However, Notch-3 was observed to be associated with lymph node metastasis (p = 0.03), increased smoking (p = 0.03), tobacco consumption (p = 0.02), vaginal involvement of tumor (p = 0.03), progressed tumor grade (p = 0.001) and FIGO stage (p = 0.03). Hence, our results reveal the possibility of Notch-3 involvement in the activation of the Notch signalling pathway in precancer and ISCC lesions. Notch-3 activation is an early event in invasive squamous carcinoma of cervix and represents a potential risk factor for poor prognosis in early-stage patients. Correlation of increased Notch-3 expression with smoking (p = 0.03) and tobacco (ST) consumption (p = 0.02) underscored its significance in ST-associated cervical carcinogenesis. Additionally, we identified that the association of Notch-3 with lymph node involvement highlights the clinical utility in ISCC. The above results also signifies that up-regulated Notch-3 and down-regulated Notch-1 expression are correlated with late clinical stage of ISCC and associated with aggressive tumor behaviour and cancer progression underscoring their potential as a candidate predictive markers for disease progression.

High sensitivity (99%, 83%; 81.6%, 84.7%) and specificity (95%, 75%; 87.5%, 87.5%) of both Notch-1 and Notch-3 in precancer and ISCC strongly supports their clinical utility as specific biomarkers for early detection of ISCC progression of cervical cancer.

Hence, this study has identified Notch-1 and Notch-3 as biomarkers that could detect the disease early, predict aggressive behavior, and define markers for more effective targeted therapy. In the near future these markers will be certainly validated, and the use of proteomics might help greatly clinicians in cancer management. The possibility of validating potential tumor markers using IHC has clear advantages as it is sensitive, easy and cost effective and virtually every pathology laboratory could perform it.

Currently, two successful prophylactic HPV vaccines-quadrivalent ‘Gardasil’ (HPV-16/18/6/11) developed by Merck while bivalent ‘Cervarix’ (HPV-16/18) by Glaxo SmithKline (GSK) are recommended for vaccinating young adolescent girls at or before onset of puberty. These two vaccines protect from infection with two of the most common cancer-causing HPV types 16/18 and in India more than 70% of cervical cancer cases are associated with these two HPV types [1]. Despite availability of two prophylactic HPV vaccines, it is difficult to control HPV infection through them. Although prophylactic vaccines appear to be successful, it would take decades to perceive the benefits because it takes several years to develop histopathologically well characterized precursors and cancerous lesions. Therefore, attempts are being made to develop therapeutic vaccines by targeting both HPV E6 and E7 oncoproteins which will serve as a bridge for temporal deficit by attacking already persistent HPV infections and to prevent cervical cancer in women [49].

The article "Clinical Impact of De-Regulated Notch-1 and Notch-3 in the Development and Progression of HPV-Associated Different Histological Subtypes of Precancerous and Cancerous Lesions of Human Uterine Cervix" was retracted in 2022. Reasons: errors in the images; duplicated images; unreliable results or conclusions.

Successful treatment of any cancer starts from early and accurate detection, confirmation, and staging of the tumor. After failure of the traditional antineoplastic drugs, targeted therapies on signalling pathways with more promise and lesser toxicity are being explored in various cancers. Activation of Wingless-related integration site (Wnt), Hedgehog (Hh) and Notch signalling is implicated in the development and progression of several tumors. Targeting these signalling pathways could therefore be a potential option for the treatment of cancers [50].

Currently, treatment of cervical cancer depends on the biopsy results (either persistent LSIL or HSIL, or invasive cancer). Other possible therapeutic modalities are both ablative (laser and cryosurgery) and excisional (cold knife conization, laser conization, loop electrocautery excision, and hysterectomy). For effective therapeutic intervention of HPV and to prevent cervical cancer development at an early stage, it is essential to improve understanding of molecular pathways involved in HPV-induced cervical carcinogenesis. The Notch pathway has tremendous potential as a new target in cancer therapy. Preclinical data evaluating the combination of inhibitors of this pathway also seem to be very promising. Notch inhibition in cancer cells has the potential to slow cell proliferation, cause apoptosis, induce differentiation and possibly trigger other terminal cell fates such as senescence. Promising results have also been obtained using various approaches including expression of Notch-1 ectodomain to inhibit tumor growth and angiogenesis [51], inhibiting γ-secretases and the ADAM metalloproteases that perform key activating cleavages of Notch [52], expressing dominant-negative fragments of Mastermind to modulate Notch signalling [51]. Notch specific γ-secretase inhibitors have also been found to prevent Notch-3 activation and to reduce proliferation in human ovarian and lung cancers [53] and in Kaposi's sarcoma [54]. Although these approaches show great potential for therapeutic intervention of Notch signalling in future, they also highlight the need for a better understanding the role of each Notch paralogue in cervical cancer, the degree to which Notch activation is triggered by distinct ADAM enzymes and γ-secretase complexes, and the extent to which inhibition of one Notch paralogue can be compensated by up-regulaton or re-expression of other Notch paralogues. Other alternatives for Notch inhibition includes: use of a stapled peptide to block interaction of Mastermind-like with the Notch intracellular domain [55], delivery of RNA interference, either small interfering RNAs (siRNAs) or endogenous or artificial microRNAs. The microRNA miR-326, miR-34a, miR-206 have been shown to target Notch-1, Notch-2 and Notch-3 to decrease the Notch activity in brain tumors [56]–[57]. Even if Notch inhibitors alone do not yield major responses and cures, there is a growing evidence that synergy can result from combining Notch inhibition with already existing treatment modalities such as chemotherapy, radiation and other pathway inhibitors to maximize their effects [58]–[59]. However, these approaches have not yet been translated into the clinic.

The article "Clinical Impact of De-Regulated Notch-1 and Notch-3 in the Development and Progression of HPV-Associated Different Histological Subtypes of Precancerous and Cancerous Lesions of Human Uterine Cervix" was retracted in 2022. Reasons: errors in the images; duplicated images; unreliable results or conclusions.

In the view of above, it is clear that biomarker studies on Notch-associated cancers aid to understand the other cellular events and signalling pathway interactions, contributing to tumor progression and further will guide the selection of the most effective therapeutic approach. Finally, it should be noted that Notch-targeting therapies are relevant not only for cancer, but also potentially for a host of developmental, vascular, cardiac, and other diseases associated with Notch pathway malfunction. The current study indicates that Notch-3 is required for proliferation and survival of Notch-3 amplified tumors and inactivation of Notch-3 is sufficient to abolish the neoplastic phenotype. Hence, detection of nuclear Notch-3 expression in cervical cancers may identify patients who may benefit from Notch inhibitors in addition to conventional cytotoxic chemotherapy or radiation therapy. This may have a potential therapeutic implication due to which Notch-3 may not trigger E6 and E7 oncoproteins of HPV to promote tumor formation in early and late stages of cervical cancer.

Notch signalling also plays critical role in cancer stem cells (CSCs). Since current cancer therapeutics do not usually target CSCs but they only kills differentiated tumor cells that make up the bulk of the tumor, thus killing of rare CSC population is of paramount importance, which could be accomplished by Notch-targeted therapy. Therefore eradication of CSCs by such novel approaches is increasingly being recognized as an important goal for the complete eradication of tumors [60].

In the view of all above, we conclude that the Notch signalling pathway, which has been exhibited to be necessary for several biological processes like cellular proliferation, differentiation, apoptosis and regulation of the cell cycle, plays critical role in the pathogenesis of HPV associated cervical cancer. The altered expression levels of its receptors- Notch-1 and Notch-3 leads to abnormal activation of this pathway. As a consequence, resulting in inappropriate signalling in HPV associated cervical cancer. This study also supports the clinical utility of these Notch receptors as specific biomarkers for early detection of ISCC. And such a unified approach may not only provide the basis for the identification of high risk premalignant lesions but may also provide potential therapeutic targets in order to control their expression levels (46). Notch inhibition may be applicable as monotherapy, or in combination with other therapies for the treatment of ISCC. However, more research into the exact mechanisms involved in Notch signalling is needed to gain more insight in the potential benefit of Notch-targeted therapy for cervical cancer treatment. Moreover, more studies are needed to investigate possible interactions of the combined modalities.

The article "Clinical Impact of De-Regulated Notch-1 and Notch-3 in the Development and Progression of HPV-Associated Different Histological Subtypes of Precancerous and Cancerous Lesions of Human Uterine Cervix" was retracted in 2022. Reasons: errors in the images; duplicated images; unreliable results or conclusions.

## Supporting Information

Figure S1 Associations between Notch Proteins in Pre-cancer and ISCC patients.
(TIF)

Table S1 Test Performance of Notch-1 (nuclear& cyto) protein in precancer and ISCC.
(DOC)

Table S2 Test Performance of Notch-3 (nuclear& cyto) protein in precancer and ISCC.
(DOC)

Table S3 Demographic characteristics and HPV status of ISCC cases, investigated from North Indian population.
(DOC)

Table S4 Correlation of HPV-16 infection with Notch-1 protein expression in CIN-1 and CIN2/3.
(DOC)

Table S5 Correlation of HPV-16 infection with Notch-3 protein expression in CIN-1 and CIN2/3.
(DOC)
